This article has been retracted.

# Intra-articular Injections With Either Triamcinolone Hexacetonide, Stanozolol, Hylan G-F 20, or a Platelet Concentrate Improve Clinical Signs in Police Working Dogs With Bilateral Hip Osteoarthritis

**DOI:** 10.3389/fvets.2020.609889

**Published:** 2021-01-18

**Authors:** João C. Alves, Ana Santos, Patrícia Jorge, Catarina Lavrador, L. Miguel Carreira

**Affiliations:** ^1^Divisão de Medicina Veterinária, Guarda Nacional Republicana (GNR), Lisbon, Portugal; ^2^MED - Mediterranean Institute for Agriculture, Environment and Development, Instituto de Investigação e Forma Avana, Universidade de Évora, Évora, Portugal; ^3^Faculty of Veterinary Medicine, University of Lisbon, Lisbon, Portugal; ^4^Interdisciplinary Centre for Research in Animal Health (CIISA), University of Lisbon, Lisbon, Portugal; ^5^Anjos of Assis Veterinary Medicine Centre (CMVAA), Barreiro, Portugal

**Keywords:** animal model, osteoarthritis, pain, intra-articular, platelet, triamcinolone, hylan G-F 20

## Abstract

**Objectives:** To compare the effect of intra-articular treatment with triamcinolone hexacetonide (TH), stanozolol, hyaluronan, and a platelet concentrate in police working dogs with bilateral hip osteoarthritis (OA).

**Study Design:** Prospective, longitudinal, double-blinded, negative controlled study.

**Sample Population:** Fifty police working dogs with naturally occurring hip OA.

**Methods:** Animals were randomly assigned to a control group (CG, *n* = 10), TH group (THG, *n* = 10), platelet concentrate group (PCG, *n* = 10), stanozolol group (SG, *n* = 10), and Hylan G-F 20 group (HG). On days 0 (T0), 8, 15, 30, 90, and 180 days post-treatment, weight-bearing distribution was evaluated. In those days, and on days 60, 120, and 150, four clinical metrology instruments were completed. Kaplan–Meier estimators were conducted and compared with the log-rank test. Cox proportional hazard regression analysis was performed to determine treatment survival. Significance was set at *p* < 0.05.

**Results:** Patients had a mean age of 6.5 ± 2.4 years and body weight of 26.7 ± 5.2 kg. At T0, hips were classified as mild (*n* = 35), moderate (*n* = 10), and severe (*n* = 5), according to the Orthopedic Foundation for Animals grading scheme. No differences were found between groups at that moment considering age, body weight, OFA hip score, and all assessments performed. All treatments improved clinical signs in various OA dimensions in some groups, with a broad effect interval. PCG showed a lower range of variation while maintaining a positive result for more extended periods (*p* < 0.01 for symmetry index and 0.01 < *p* < 0.04 in the majority of scores). Breed, age, sex, and OFA grade did not significantly influence response to treatment.

**Conclusions and Clinical Relevance:** This is the first prospective, negative controlled, double-blinded study to compare the effect of a single administration of these IA treatments in dogs with hip OA. HG and PCG recorded more significant improvements throughout the 180-day follow-up. In particular, PCG also registered a lower variation in results, seemingly the best therapeutic option. Nevertheless, improvements were still observed in THG and SG, and these treatment options can be considered, mainly when the first two treatments are not available.

## Introduction

Osteoarthritis (OA) is the most commonly diagnosed joint disease in veterinary medicine, with at least 80% of the cases of lameness and joint diseases in companion animals broadly classified as OA (1–3). Risk factors for developing OA are well documented and include breed, neutering, higher body weight, and age > 8 years (4). For the evaluation of hip OA, pelvic radiographs are frequently performed (5–7). Weight distribution, off-loading, or limb favoring at stance is a commonly used subjective assessment during orthopedic examination (8). Animals with OA may not be overtly lame but exhibit subtle shifts in body weight distribution at a stance due to pain or instability, which are detectable with force plate gait analysis and weight distribution platforms (9, 10). Body weight distribution at a stance may even be an equivalent or superior measurement of pain associated with hip OA than vertical impulse or peak vertical force (10, 11). Pain is a hallmark of OA, affecting more than just the functional aspect of the disease, and the evaluation of treatment success should encompass the assessment of these multiple dimensions of OA (12, 13). Clinical metrology instruments (CMIs) aim to evaluate multiple dimensions of OA, and the commonly used instruments in dogs are the Canine Brief Pain Inventory (CBPI, divided into a pain severity score—PSS, and a pain interference score—PIS) and the Liverpool Osteoarthritis in Dogs (LOAD) (12, 14–20). Additional validated CMIs include the Hudson Visual Analog Scale (HVAS), a valid tool to assess the degree of lameness in dogs, with force plate analysis as a criterion-referenced standard, and the Canine Orthopedic Index (COI, divided into four scores: stiffness, gait, function, and quality of life—QOL) (21–23).

The medical approach to OA aims at slowing disease progression, relieving pain, and improving overall function (14, 24), and it is well suited to be addressed through the use of local therapy by intra-articular (IA) injection (25, 26). IA corticosteroids have been used for several decades. Currently, different guidelines for the management of human OA provide varying strength of recommendation for the use of IA corticosteroids, from weak to strong recommendation (27–31). Some reports present deleterious effects of IA corticosteroids, namely, the induction of a low-quantity and high-viscosity synovial fluid. These results are often based on multiple injections, particularly of methylprednisolone, while a single dose does not seem to cause long-term detrimental effects (32, 33). Triamcinolone hexacetonide (TH), in particular, can provide pain relief, improve mobility for prolonged periods, and reduce the severity of structural changes (28, 34–36). Hyaluronan is also a commonly used treatment modality in OA management, although its action mechanism is not entirely known (37, 38). It has been proposed to have anti-inflammatory, anti-nociceptive, and chondroprotective properties (39–42). High-molecular-weight products seem to produce better results (43–46). Autologous platelets are a regenerative treatment modality for OA, acting through a supraphysiologic release of growth factors directly at the treatment site, promoting tissue regeneration and attraction of mesenchymal stem cells (47–50). In dogs, a single IA PRP (platelet-rich plasma) injection has resulted in clinical improvements for 12 weeks in some reports, and up to 6 months according to others. In some cases, these improvements occur without the progression of radiographic signs (51–54).

Multiple injection protocols have also been described, producing a positive effect on joint range of motion, pain, lameness, and kinetics (55). More recently, the use of stanozolol, a synthetic derivative of testosterone, has been described in animal models. When administered IA, it induced fibroblasts to increase collagen production, decrease nitric oxide production, and induce osteoblast proliferation and collagen synthesis. It also has a chondroprotective and cartilage regeneration effect while reducing osteophyte formation and subchondral bone reaction (56–61).

To compare long-term outcomes and to identify factors associated with response to treatment, we compared the effect of the IA administration of TH, Hylan G-F 20, stanozolol, and a platelet concentrate in the treatment of police working dogs with bilateral hip OA. We hypothesize that the different treatments will be able to improve CMIs scores and weight-bearing distribution in dogs with OA, compared to a control group (CG).

## Methods

The study protocol was approved by the ethical review committee of the University of Évora (Órgão Responsável pelo Bem-estar dos Animais da Universidade de Évora, approval no GD/32055/2018/P1, September 25, 2018). Written informed consent was obtained from the institution responsible for the animals. Fifty active police working dogs with bilateral hip OA were selected to participate in this prospective, longitudinal, double-blinded, negative controlled study. They were included based on history, physical, orthopedic, neurological, and radiographic examinations compatible with bilateral hip OA. Hips were classified according to the Orthopedic Foundation for Animals hip grading scheme at the initial evaluation, on day 0 (62, 63). Animals suspected or with any other orthopedic, or concomitant disease (ruled out through physical examination, complete blood count, and serum chemistry profile) were excluded. Additionally, animals were >2 years old, weighed >20 kg and had no other medications or nutritional supplements administered for the previous 6 weeks and during the study period. Patients were randomly assigned to five different groups, using the statistical analysis software, according to the treatment being administered: a CG (*n* = 10), receiving an IA administration of 2 ml of NaCl 0.9% per hip joint; a triamcinolone hexacetonide group (THG, *n* = 10), receiving 20 mg/ml of TH (Bluxam, Riemser Pharma, Portugal) per hip joint; a platelet concentrate group (PCG, *n* = 10), which received 3 ml of platelet concentrate per hip joint; a stanozolol group (SG, *n* = 10), to which 0.3 mg/kg of stanozolol (Estrombol, Laboratório Fundacion) per hip joint (64, 65) was administered; and a hyaluronan group (HG, *n* = 10), which received 2 ml of Hylan G-F 20 (Synvisc®, Sanofi, Portugal) per hip joint. All treatments were administered only on day 0 (treatment day) through IA administration. According to the manufacturer's instructions, this specific platelet concentrate was prepared with the commercially available kit (V-PET®, PALL Corporation). Briefly, 55 ml of whole blood was collected from the jugular vein and introduced into the provided closed system for its preparation. The blood was then allowed to flow by gravity through a filter, where the platelets were concentrated. The platelet concentrate was then recovered and administered within 5 min of preparation.

All IA administrations and radiographic examinations were conducted under light sedation, obtained with the simultaneous intravenous administration of medetomidine (0.01 mg/kg) and butorphanol (0.1 mg/kg). For IA administrations, patients were placed in lateral recumbency with the treatment joint dorsal. The anatomical reference for access was the greater trochanter, around which a 4 × 4 cm window was clipped and aseptically prepared. After preparation, an assistant placed the limb in a neutral position, parallel to the table. A 21-gauge with 2.5 length needle was then introduced just dorsal to the greater trochanter, perpendicular to the limb's long axis until the joint was reached (66). Confirmation of correct needle placement was obtained by collecting synovial fluid, withdrawing as much synovial fluid as possible, and the respective substance was administered. Ultrasound guidance was available if required to confirm the correct needle placement. After treatment, animals were rested for three consecutive days and examined by a veterinarian on days 1 and 3 post procedure to determine signs of exacerbated pain, persistent stiffness of gait, and posture changes. If no complaints were registered, the animal was allowed to resume its normal activity (54, 67). On days 0, 8, 15, 30, 90, and 180 post-treatment, weight distribution was conducted with a stance analysis platform (Companion Stance Analyzer; LiteCure LLC, Newark, Delaware, United States), placed in the center of a room, at least 1 m from the walls. It was calibrated at the beginning of each testing day and zeroed before each data collection. Animals stood on the platform, with one foot on each quadrant of the platform, while maintaining a natural stance with their center of gravity near the platform's middle. When required, gentle restraint was used to maintain the patient's head in a natural forward-facing position. The left–right symmetry index (SI) was calculated according to the following formula: SI = [(WB_R_ – WB_L_)/((WB_R_ + WB_L_) × 0.5)] × 100, where WB_R_ is the value of weight-bearing for the right pelvic limb and WB_L_ is the value of weight-bearing for the left pelvic limb. Negative values were made positive (19, 68). Since all animals included in the study had bilateral disease, we also considered a deviation from the normal 40% weight-bearing for the combined pelvic limbs (10), calculated by subtracting WB to the normal 40%_._ On days 0, 8, 15, 30, 60, 90, 120, 150, and 180 post-treatment after treatment, an online copy of the HVAS, CBPI, COI, and LOAD was completed by the dogs' trainers after receiving the published instructions for each of them. Dogs' trainers were unaware of which treatment the animal received. The CMIs were completed in sequence by the same handler in all follow-up moments, without knowing their previous answer. The two sections of the CBPI (PSS and PIS) and COI's four dimensions (stiffness, function, gait, and QOL) were considered separately in the analysis. All evaluations were performed at the same moment by the same researcher blinded to the group and identity of the patient.

For the considered IA treatments, some side effects are documented and include local pain and local inflammation. These are usually self-limiting and take 2–10 days to resolve (69). The occurrence of these side effects was monitored during treatment follow-up assessments and recorded.

Demographic data as age, sex, body weight, and breed were recorded. Kaplan–Meier estimators were conducted to generate survival curves and survival probability and compared with the log-rank test. Cox proportional hazard regression analysis was carried out to investigate interest variables' influence (age, sex, body weight, breed, and OFA score) on survival. All results were analyzed with IBM SPSS Statistics version 20, and a significance level of *p* < 0.05 was set. With the CBPI, a specific measure of success was defined and set as a reduction of ≥1 in PSS and ≥2 in PIS (70). The time for PIS and PSS scores to drop below the defined level of reduction was evaluated. For the remaining CMIs scores and weight-bearing evaluation, the outcome considered was a return to or drop below values recorded at the initial evaluation. Patients with values or scores above baseline values at the evaluation moment the event was recorded were censored.

## Results

The sample included 50 police working dogs, of both genders (30 males and 20 females), with a mean age of 6.5 ± 2.4 years and body weight of 26.7 ± 5.2 kg. Four dog breeds were represented: German Shepherd Dogs (GSD, *n* = 17), Belgian Malinois Shepherd Dogs (BM, *n* = 15), Labrador Retriever (LR, *n* = 10), and Dutch Shepherd Dogs (DSD, *n* = 8). Considering OFA hip grading, 35 animals were classified as mild (70%), 10 were classified as moderate (20%), and 5 were classified as severe (10%). The platelet concentrate obtained had a four-fold platelet concentration, a two-fold leukocyte concentration, and a 50% reduction in platelet concentrate hematocrit than whole blood values. These values are in line with those previously described for V-PET® (71). The results of the evaluation performed at day 0, by group, are presented in Table 1, where no significant differences were found between groups. Results of the Kaplan–Meier estimators are presented in Table 2. All treatments were able to produce better results than CG, with variable periods of duration. Better results were observed in the PCG and HG in all considered outcome measures, with a lower range with a 95% confidence interval. Results of the Cox proportional hazard regression are presented in Table 3. Treatment was the covariable that contributed more frequently to the outcomes observed. In fact, in some cases (as SI, HVAS, PIS, and others), it was the only one. Only overall COI also influenced the OFA score, with dogs with a severe hip grade having a 4.1-fold probability of returning to baseline values, compared with dogs with a mild grade. LOAD was the only outcome measure influenced by breed, with DSD showing a lower risk baseline values. All patients were followed up to the 180-day evaluation moment. Post-injection increased lameness was observed in eight patients in PCG, four in SG, three in HG, and two in THG, which spontaneously resolved within 48–72 h. No additional treatment or medications was administered to the animals during this period.

**Table 1:** Mean values (± standard deviation) at initial evaluation of evaluation conducted for control and treatment groups.

**Treatment group**	**Age**	**Weight (kg. mean ± SD)**	**Symmetry Index (mean ± SD)**	**Deviation (mean ± SD)**	**HVAS (0–10)**	**PSS (0–10)**	**PIS (0–10)**	**LOAD (0–52)**	**Stiffness (0–16)**	**Function (0–16)**	**Gait (0–20)**	**QOL (0–12)**	**COI (0–64)**
CG	6.5 ± 2.5	28.3 ± 5.4	33.6 ± 24.3	2.1 ± 1.8	7.2 ± 0.9	2.4 ± 1.5	2.5 ± 1.7	12.3 ± 8.3	3.1 ± 2.9	3.1 ± 3.5	4.1 ± 4.0	3.6 ± 2.5	13.9 ± 12.6
THG	6.0 ± 2.6	27.4 ± 6.0	41.7 ± 41.7	4.4 ± 3.3	6.2 ± 1.7	3.2 ± 2.4	3.8 ± 2.9	18.2 ± 12.6	5.1 ± 3.9	4.3 ± 5.0	7.6 ± 5.8	4.6 ± 3.6	21.6 ± 17.7
HG	7.2 ± 2.6	26.5 ± 3.2	20.3 ± 21.8	5.6 ± 4.5	6.5 ± 1.4	3.3 ± 2.4	3.3 ± 2.2	16.6 ± 10.4	3.5 ± 3.1	4.5 ± 3.5	7.1 ± 4.7	4.7 ± 2.8	19.8 ± 12.7
SG	5.5 ± 1.9	26.0 ± 2.9	24.5 ± 13.2	6.0 ± 5.6	6.6 ± 1.3	2.3 ± 1.7	2.3 ± 1.6	8.2 ± 5.1	3.6 ± 2.4	1.1 ± 1.7	3.3 ± 3.9	3.1 ± 2.2	16.1 ± 16.5
PCG	7.1 ± 1.9	27.4 ± 6.3	21.0 ± 11.6	4.8 ± 2.3	6.4 ± 1.0	2.7 ± 2.3	2.7 ± 2.5	12.3 ± 9.6	3.3 ± 3.1	3.6 ± 4.5	4.6 ± 4.9	4.5 ± 3.3	16.0 ± 14.7

*CG, Control group; COI, Canine Orthopedic Index; HG, Hylan G-F 20 group; HVAS, Hudson Visual Analog Scale; LOAD, Liverpool Osteoarthritis in Dogs; OFA, Orthopedic Foundation for Animals; PCG, Platelet Concentrate group; PIS, Pain Interference Score; PSS, Pain Severity Score; QOL, Quality of Life; SG, Stanozolol group; THG, Triamcinolone hexacetonide group*.

**Table 2:** Survival probability calculated with Kaplan-Meier estimators (in days) and compared with the log rank test.

		**Treatment**									
**Variable**	**Log rank test**	**CG**		**HG**		**PCG**		**SG**		**THG**	
		**Mean ± SD**	**95% CI**	**Mean ± SD**	**95% CI**	**Mean ± SD**	**95% CI**	**Mean ± SD**	**95% CI**	**Mean ± SD**	**95% CI**
Symmetry Index	0.000^*^	28.6 ± 7.5	13.9–43.2	111.8 ± 20.5	71.5–152.1	171.0 ± 9.5	152.3–189.7	80.3 ± 19.6	43.7–116.9	94.5 ± 16.8	78.8–115.7
Deviation	0.031^*^	48.8 ± 16.6	16.3–81.3	130.5 ± 22.3	86.8–174.2	147.0 ± 18.6	110.5–183.5	90.8 ± 23.9	43.8–137.8	99.0 ± 23.7	52.5–145.5
HVAS	0.012^*^	49.7 ± 17.5	15.4–84.0	117.0 ± 18.7	80.3–153.7	144.0 ± 17.3	110.2–177.8	129.8 ± 18.9	92.7–166.9	66.1 ± 20.1	26.7–105.5
PSS	0.485	63.2 ± 24.3	15.6–110.8	142.5 ± 16.9	109.4–175.7	150.0 ± 14.3	122.1–177.9	94.6 ± 23.2	49.2–140.0	90.2 ± 24.9	41.4–139.0
PIS	0.000^*^	8.7 ± 0.7	7.3–10.1	114.0 ± 22.7	69.6–158.4	138.0 ± 15.8	106.9–169.1	109.6 ± 25.6	59.4–159.8	118.6 ± 23.0	76.5–119.0
LOAD	0.000^*^	40.7 ± 16.3	10.6–70.8	141.8 ± 16.3	109.8–173.8	120.0 ± 18.7	83.3–156.6	123.8 ± 20.1	84.5–163.1	124.3 ± 22.5	80.2–129.4
Stiffness	0.592	64.7 ± 24.0	17.7–111.7	129.8 ± 20.5	89.7–169.9	141.0 ± 15.7	110.1–171.9	111.8 ± 22.5	67.7–155.9	130.8 ± 16.4	98.7–162.9
Function	0.013^*^	65.4 ± 18.9	28.4-102.4	168.0 ± 10.0	148.3–187.7	135.0 ± 13.8	107.9–162.0	124.5 ± 21.8	81.7–167.3	112.6 ± 22.1	69.3–155.9
Gait	0.328	52.7 ± 20.7	12.1–93.3	115.5 ± 18.5	79.2–151.8	123.0 ± 18.3	87.2–158.8	103.6 ± 26.2	60.0–147.2	117.0 ± 22.2	73.5–160.5
QOL	0.533	60.9 ± 21.3	19.2–102.6	120.0 ± 17.5	85.7–154.3	120.8 ± 19.2	83.1–158.5	66.2 ± 25.7	15.9–116.5	119.3 ± 25.8	68.8–169.8
COI	0.380	52.7 ± 18.9	15.7–89.7	93.1 ± 23.6	46.8–139.4	138.0 ± 15.7	107.2–168.8	78.1 ± 19.8	39.3–116.9	78.9 ± 22.5	34.8–123.0

*CG, Control group; COI, Canine Orthopedic Index; HG, Hylan G-F 20 group; HVAS, Hudson Visual Analog Scale; LOAD, Liverpool Osteoarthritis in Dogs; OFA, Orthopedic Foundation for Animals; PCG, Platelet Concentrate group; PIS, Pain Interference Score; PSS, Pain Severity Score; QOL, Quality of Life; SG, Stanozolol group; THG, Triamcinolone hexacetonide group*.

* *indicates significance*.

**Table 3:** Results Cox proportional hazard regression with the different outcome evaluations.

	**Weight distribution**						**CBPI**					
**Variable**	**Symmetry Index (*****p*** **=** **0.014)**		**Deviation (*****p*** **=** **0.251)**		**HVAS (*****p*** **=** **0.036)**		**PSS (*****p*** **=** **0.881)**		**PIS (*****p*** **=** **0.025)**		**LOAD (*****p*** **=** **0.006)**	
	**HR (95% CI)**	***p***	**HR (95% CI)**	***p***	**HR (95% CI)**	***p***	**HR (95% CI)**	***p***	**HR (95% CI)**	***p***	**HR (95% CI)**	***p***
**Treatment**		0.001^*^		0.159		0.005^*^		0.529		0.001^*^		0.000^*^
Control	1.00		1.00		1.00		1.00		1.00		1.00	
HG	0.23 (0.08–0.65)	0.006^*^	0.25 (0.07–0.84)	0.026^*^	0.19 (0.06–0.64)	0.007^*^	0.29 (0.08–1.16)	0.081	0.06 (0.15–0.26)	0.000^*^	0.06 (0.02–0.25)	0.000^*^
PCG	0.24 (0.21–0.26)	0.000^*^	0.29 (0.09–0.96)	0.042^*^	0.26 (0.09–0.82)	0.021^*^	0.57 (0.19–1.73)	0.322	0.12 (0.03–0.43)	0.001^*^	0.19 (0.06–0.62)	0.005^*^
SG	0.21 (0.07–0.60)	0.004^*^	0.42 (0.12–1.47)	0.176	0.31 (0.09–1.08)	0.066	0.65 (0.19–2.18)	0.487	0.09 (0.02–0.36)	0.001^*^	0.08 (0.02–0.28)	0.000^*^
THG	0.29 (0.09-0.83)	0.021^*^	0.53 (0.18–1.54)	0.245	0.58 (0.20–1.66)	0.311	0.72 (0.23–2.25)	0.573	0.08 (0.02–0.32)	0.000^*^	0.09 (0.03–0.36)	0.001^*^
**OFA score**		0.582		0.608		0.195		0.998		0.621		0.211
Mild	1.00		1.00		1.00		1.00		1.00		1.00	
Moderate	0.70 (0.29–1.69)	0.430	0.75 (0.30–1.85)	0.528	1.49 (0.63–3.52)	0.358	1.024 (0.41-2.57)	0.960	1.53 (0.65–3.61)	0.330	2.18 (0.89–5.34)	0.088
Severe	0.58 (0.17–1.94)	0.378	1.44 (0.37–5.58)	0.597	3.00 (0.88–10.29)	0.079	0.99 (0.22–4.41)	0.990	1.25 (0.31–5.00)	0.749	1.03 (0.23–4.61)	0.972
**Breed**		0.861		0.293		0.752		0.856		0.631		0.073
LR	1.00		1.00		1.00		1.00		1.00		1.00	
GSD	0.74 (0.24–2.28)	0.589	0.44 (0.13–1.54)	0.202	0.52 (0.13–2.14)	0.368	1.42 (0.36–5.61)	0.619	0.52 (0.14–1.92)	0.327	0.76 (0.21–2.76)	0.672
BM	0.63 (0.21–1.91)	0.411	0.31 (0.09–1.13)	0.076	0.47 (0.12–1.85)	0.283	0.92 (0.27–3.15)	0.888	0.46 (0.14–1.58)	0.217	0.35 (0.09–1.33)	0.121
DSD	0.79 (0.22–2.86)	0.724	0.58 (0.12–2.74)	0.493	0.58 (0.13–2.72)	0.493	1.39 (0.54–2.92)	0.684	0.43 (0.10–1.82)	0.249	0.17 (0.03–0.83)	0.028^*^
**Sex**												
Male	1.00		1.00		1.00		1.00		1.00		1.00	
Female	1.51 (0.76–2.99)	0.238	0.77 (0.34–1.75)	0.536	0.33 (0.12–0.87)	0.025^*^	1.25 (0.54–2.92)	0.607	0.85 (0.37–1.97)	0.704	1.17 (0.49–2.79)	0.721
**Age**	0.90 (0.77–1.06)	0.216	0.9 (0.75–1.09)	0.274	1.09 (0.91–1.29)	0.363	1.13 (0.93–1.37)	0.222	0.912 (0.77–1.08)	0.299	0.9 (0.76–1.07)	0.229
	**COI**												
**Variable**	**Stiffness (*****p*** **=** **0.034)**		**Function (*****p*** **=** **0.023)**			**Gait (*****p*** **=** **0.069)**			**QOL (*****p*** **=** **0.325)**		**Total (*****p*** **=** **0.053)**	
	**HR (95% CI)**	***p***	**HR (95% CI)**		***p***		**HR (95% CI)**	***p***	**HR (95% CI)**	***p***	**HR (95% CI)**	***p***
**Treatment**		0.099			0.022^*^			0.056		0.840		0.163
Control	1.00		1.00				1.00		1.00		1.00	
HG	0.19 (0.05–0.74)	0.016^*^	0.09 (0.02–0.43)		0.002^*^		0.20 (0.06–0.71)	0.012^*^	0.64 (0.19–2.09)	0.463	0.29 (0.09–0.92)	0.036^*^
PCG	0.23 (0.07–0.77)	0.018^*^	0.33 (0.11–1.02)		0.054		0.21 (0.07–0.67)	0.009^*^	0.57 (0.21–1.58)	0.282	0.29 (0.09–0.87)	0.030^*^
SG	0.31 (0.09–1.09)	0.069	0.28 (0.08–1.01)		0.051		0.36 (0.11–1.15)	0.083	0.87 (0.28–0.67)	0.807	0.54 (0.17–1.66)	0.279
THG	0.31 (0.09–1.09)	0.069	0.33 (0.11–1.02)		0.054		0.29 (0.09–0.92)	0.036^*^	0.65 (0.22–1.96)	0.444	0.49 (0.17–1.41)	0.188
**OFA score**		0.223			0.068			0.439		0.303		0.041^*^
Mild	1.00		1.00				1.00		1.00		1.00	
Moderate	1.05 (0.39–2.84)	0.918	0.89 (0.34–2.36)		0.823		0.63 (0.24–1.64)	0.344	0.48 (0.19–1.22)	0.123	0.69 (0.28–1.73)	0.431
Severe	3.11 (0.79–12.13)	0.102	5.09 (1.18–21.98)		0.029^*^		1.34 (0.39–4.629	0.641	0.78 (0.22–2.77)	0.696	4.19 (1.08–16.24)	0.038^*^
**Breed**		0.069			0.559			0.255		0.320		0.997
LR	1.00		1.00				1.00		1.00		1.00	
GSD	0.46 (0.10–2.00)	0.298	2.54 (0.56–11.47)		0.226		0.71 (0.18–2.78)	0.622	2.31 (0.65–8.25)	0.199	0.92 (0.26–3.28)	0.898
BM	1.39 (0.40–4.81)	0.606	2.04 (0.52–7.99)		0.309		1.15 (0.33−3.96)	0.824	0.87 (0.33–7.49)	0.814	0.92 (0.29–2.93)	0.893
DSD	0.22 (0.03–1.51)	0.124	1.18 (0.22–6.22)		0.845		0.29 (0.05–1.58)	0.153	1.57 (0.33–7.49)	0.572	1.00 (0.24–4.15)	0.995
**Sex**												
Male	1.00		1.00				1.00		1.00		1.00	
Female	1.49 (0.60–3.69)	0.386	1.58 (0.62–4.01)		0.337		1.19 (0.52–2.74)	0.685	3.16 (1.35–7.39)	0.008^*^	2.02 (0.89–4.55)	0.089
**Age**	1.08 (0.91–1.29)	0.378	1.16 (0.96–1.41)		0.119		1.19 (0.99–1.43)	0.071	1.06 (0.87–1.29)	0.572	1.14 (0.94–1.37)	0.180

*BM, Belgian Malinois Shepherd Dog; CBPI, Canine Brief Pain Inventory; COI, Canine Orthopedic Index; DSD, Dutch Shepherd Dog; GSD, German Shepherd Dog; HG, Hylan G-F 20 group; HVAS, Hudson Visual Analog Scale; LOAD, Liverpool Osteoarthritis in Dogs; LR, Labrador Retriever; OFA, Orthopedic Foundation for Animals; PCG, Platelet Concentrate group; PIS, Pain Interference Score; PSS, Pain Severity Score; QOL, Quality of Life, SG, Stanozolol group; THG, Triamcinolone hexacetonide group*.

* *indicates significance*.

## Discussion

OA is a chronic disease with no cure. Therefore, the main focus of OA management is to control clinical signs, mainly pain levels (72, 73). Hip OA, in particular, is very common in large breed dogs such as German Shepherd Dogs and Labradors. It has a toll on the quality of life, particularly in working dogs, to whom it also affects performance (74, 75). To our knowledge, this is the first prospective, negative controlled, double-blinded study to compare the long-term effects of these different IA approaches for the management of dogs with bilateral hip OA.

Clinical presentation of patients with OA is characterized by variable degrees of clinical and functional impairments. It is well established that clinical signs and the severity of pain, in particular, correlate with the functional status rather than radiographic grading of OA. For that reason, treatment should be planned according to clinical features and functional status instead of radiological findings (62, 76–78). With that in mind, we evaluated the impact of predisposing and clinical factors of OA as demographic characteristics of interest. The IA TH administration has been described as having long-term safety while improving the joint range of motion and pain compared with saline injection (79–82).

Similarly, IA hyaluronan improves pain, function, lameness, and kinetics compared to pre-treatment and saline control in patients with OA (69). Reports of canine OA treatment with this same platelet concentrate present improvements in pain, kinetics, and joint range of motion, lasting from 12 weeks to 6 months (52, 54). The use of IA stanozolol has been published in horses and an ovine model and presented as able to resolve signs of lameness, reduce osteophyte formation and subchondral bone reaction, and promote articular cartilage regeneration (58, 59). In the study presented here, all treatments improved clinical signs in various dimensions of OA in police working dogs with bilateral disease. While being able to do so, the 95% confidence interval was wide for those treatments in some groups. Values and scores in PCG showed a lower range of variation while maintaining a positive result for more extended periods. Except for pain scores, mean values in CG did not return to baseline values immediately at the first follow-up periods, as would possibly be expected. A functional improvement following NaCl IA injections has been described, and, in some instances, effects were noted up until 6-month post-administration (83). This fact can be associated with the removal of inflammatory mediators presented in the synovial fluid, and an effect similar to a joint lavage produced by the administration of saline (83), and may be the reason for the recorded evaluation in CG. Also noteworthy, while any treatment did not significantly influence PSS scores, PIS scores were. It is not uncommon that police working dogs do not show overt signs of pain, which is easily detected through its effect on daily activities and performance (84). Probably for that reason, all treatments were able to produce an 88–94% improvement compared to CG, as evaluated with the PSS. The weight-bearing evaluation platform has been deemed a repeatable and accessible device to measure static weight distribution, compared to a pressure-sensitive walkway (10, 85, 86). A significant improvement was observed only with SI considering the two weight-bearing evaluations evaluated. Dogs presenting with pelvic limb lameness tend to distribute weight more by side-to-side compensation than pelvic-to-thoracic (87, 88). This compensation mechanism may be the reason for this result, and the same compensation mechanism may be present in animals with bilateral disease, such as hip OA. This may be the reason for the wide ranges observed in standard deviations of the SI at the initial evaluation. Despite being a bilateral disease, it is not to say that both joints are affected equally, causing the animal to off-load one limb while supporting more weight on the contralateral limb. The degree of this compensation mechanism can vary between individual dogs. The same can be considered for the wide ranges in COI scores, since this CMI focuses on the ability of the dog to perform daily activities, and the clinical signs of OA patients can vary quite significantly (21).

Also, dogs included were active police working dogs, known to be stoic and not to show overt pain signs (75, 84). The fact that they were signaled to undergo treatment for hip may indicate that these animals were, at the time, in pain (86). With HVAS, HG and PCG registered more significant improvements throughout the 180-day follow-up, also with a lower variation with the 95% confidence interval. When using LOAD, all treatments produced improvements that ranged from 81 to 94%. When using the various dimensions of COI, PCG and HG were the treatments consistently leading to improvements. With this information in mind, and considering the variety of evaluations performed, the platelet concentrate and Hylan G-F 20 seem to be the best IA therapeutic choices for treating bilateral hip OA. Nevertheless, TH and stanozolol were also able to improve patients' condition and are valid therapeutic options that should be considered, mainly when the first two treatments are not available.

Heavier dogs are more prone to develop OA earlier in life (89, 90), and being overweight is a risk factor for OA. While being related, these two concepts are not the same. Since the animals that comprised the sample were active working dogs, with a body condition score of 4 or 5/9, none was overweight. Also, since represented dog breeds were all large, we chose not to include body weight as a possible influencing factor in our models. Age did not have a significant role in any of the evaluations performed, but increasing age, particularly over 8 years, is a predisposing factor for OA (4). This lack of effect may be attributed to the fact that the sample animals' mean age was below 8 years. It is also possible that age is not a factor by itself, and instead reflects the progression of the disease, which, in turn, may affect response to treatment. OFA grading only influenced function evaluation, with animals with a severe classification showing a significantly worse evolution than those graded as mild. Hylan G-F 20 seems to be the better therapeutic option for these patients since HG was the only group to show significant improvements compared to control. The reason for this may be related to the mechanism of action of hyaluronan, which supplements the viscosity and elasticity of synovial fluid (37). The remaining treatments act by interacting with joint cells and tissues, which may not be as responsive or even present in enough number to show a better response. Certain dog breeds are also at increased risk of developing hip OA since it is a common consequence of hip dysplasia and influenced by a wide range of breed-specific genes (polygenetic trait) (4, 62). Dog breeds included in this sample are known breeds at risk to develop OA and similar size and conformation. With the considered evaluation, no significant differences were observed regarding response to treatment.

There are recommendations for different administration frequency in human, canine, and horse reports. For corticosteroids, a period of at least 6–12 weeks should be respected between administrations, without exceeding two to four injections of the same joint within a year (91, 92). In horses, a study considering triamcinolone acetonide showed no difference between single or multiple administrations (93). For hyaluronan, some reports indicate that three injections weekly are more effective in reducing pain in humans when compared to a single administration, although both protocols improved joint function (94). For canine platelet products, two administrations 2–3 weeks apart have been recommended (52). We chose to administer a single IA inject to compare all treatments before evaluating multiple-administration protocols. Also, available canine recommendations are usually based on recommendations for other species or on data from canine surgical models, raising the need for information from dogs with naturally occurring OA. The fact that the animals enrolled in this study are working dogs means that their musculoskeletal structures are under greater demand than in a companion animal (95). While results may remain significant for a more extended time in companion animals, due to lower physical demand, most of the animals included in this study were being treated at an early age and with less radiographic changes than what is described in companion animals (4).

With all used IA treatments, some side effects are documented and include local pain and local inflammation. These are usually self-limiting and take 2–10 days to resolve, being attributed to a joint capsule expansion following the IA administration (59, 69, 96, 97). Similarly, we observed increased lameness in eight patients in PCG, four in SG, three in HG, and two in THG, which spontaneously resolved within 48–72 h. PCG was the group where the higher treatment volume was administer, which may account for higher number of increased lameness observed.

This study presents some limitations, namely, the inclusion of a majority of dogs with mild OA. For that reason, further studies should include a larger number of dogs with moderate and severe OA to determine if similar results are obtained. Still, a significant difference between mild and severe OA was observable in the COI score. Different volumes were administered in different groups, ranging from 1 ml (in THG) to 3 ml (in PCG). This difference in volumes may impact clinical signs following the administration, as a higher volume can produce joint capsule dilation and, consequently, pain. In our study, this did not significantly impacted the overall results, as this increased lameness resolved within 72 h in all groups, but is a variation to consider in future studies. Different numbers of administration should also be tested.

## Conclusions and Clinical Relevance

To our knowledge, this is the first prospective, negative controlled, double-blinded study to compare the effect of these different IA treatment modalities in police working dogs with bilateral hip OA. It describes each treatment modality's effect on pain level and functional evaluation, their duration, and relevant information regarding patient selection for each treatment. HG and PCG recorded greater improvements throughout the 180-day follow-up. In particular, PCG also registered a lower variation in results, seemingly the best therapeutic option. Improvements were still observed in THG and SG, and these treatment options can be considered, mainly when the first two treatments are not available.

## Data Availability Statement

The datasets generated for this article are not readily available because the data used in this study is a property of the Guarda Nacional Republicana, a governmental police force from Portugal and, by law, confidential. The authors obtained specific approval in order to use the data. Requests to access the datasets should be directed to the Divisão de Medicina Veterinária (ari.dsad.dmv@gnr.pt).

## Ethics Statement

This study is a part of a project approved by the ethical review committee of the University of Évora (Órgão Responsável pelo Bem-estar dos Animais da Universidade de Évora, approval no. GD/32055/2018/P1, September 25, 2018).

## Author Contributions

JA designed the protocol, conducted treatments, and prepared the manuscript. PJ and AS selected patients and conducted treatments. CL and LC revised the protocol and prepared the manuscript. All authors contributed to the article and approved the submitted version.

## Conflict of Interest

The V-PET kits used in this study were provided by the Pall Corporation and the Stance Analyser used in this study was provided by Companion, LiteCure LLC^®^. The authors declare that the research was conducted in the absence of any commercial or financial relationships that could be construed as a potential conflict of interest.

## References

[1] BlissS Musculoskeletal structure and physiology. In: Zink C, Van Dyke J, editors. Canine Sports Medicine and Rehabilitation. 2nd ed John Wiley & Sons, Ltd (Hoboken, NJ) (2018). p. 32–59.

[2] VenableROStokerAMCookCRCockrellMKCookJL. Examination of synovial fluid hyaluronan quantity and quality in stifle joints of dogs with osteoarthritis. Am J Vet Res. (2008) 69:1569–73. 10.2460/ajvr.69.12.156919046002

[3] JohnstonSAMcLaughlinRMBudsbergSC. Nonsurgical management of osteoarthritis in dogs. Vet Clin North Am Small Anim Pract. (2008) 38:1449–70. 10.1016/j.cvsm.2008.08.00118954692

[4] AndersonKLO'NeillDGBrodbeltDCChurchDBMeesonRLSarganD. Prevalence, duration and risk factors for appendicular osteoarthritis in a UK dog population under primary veterinary care. Sci Rep. (2018) 8:5641. 10.1038/s41598-018-23940-z29618832PMC5884849

[5] GordonWJConzemiusMGRiedeselEBesanconMFEvansRWilkeV. The relationship between limb function and radiographic osteoarthrosis in dogs with stifle osteoarthrosis. Vet Surg. (2003) 32:451–4. 10.1053/jvet.2003.5005114569573

[6] BudsbergSC. Outcome assessment in clinical trials involving medical management of osteoarthritis in small animals. Vet Clin North Am Small Anim Pract. (1997) 27:815–23. 10.1016/S0195-5616(97)50081-79243782

[7] JohnsonASmithCPijanowskiGHungerfordL. Triple pelvic osteotomy: effect on limb function and progression of degenerative joint disease. J Am Anim Hosp Assoc. (1998) 34:260–4. 10.5326/15473317-34-3-2609590455

[8] LascellesBDXRoeSCSmithEReynoldsLMarkhamJMarcellin-LittleD. Evaluation of a pressure walkway system for measurement of vertical limb forces in clinically normal dogs. Am J Vet Res. (2006) 67:277–82. 10.2460/ajvr.67.2.27716454633

[9] SeibertRMarcellin-LittleDJRoeSCDePuyVLascellesBDX. Comparison of body weight distribution, peak vertical force, and vertical impulse as measures of hip joint pain and efficacy of total hip replacement. Vet Surg. (2012) 41:443–7. 10.1111/j.1532-950X.2012.00957.x22548436

[10] CloughWCanappSTaboadaLDycusDLeasureC. Sensitivity and specificity of a weight distribution platform for the detection of objective lameness and orthopaedic disease. Vet Comp Orthop Traumatol. (2018) 31:391–5. 10.1055/s-0038-166706330300913

[11] LascellesBFreireMRoeSDePuyVSmithEMarcellin-LittleD. Evaluation of functional outcome after BFX total hip replacement using a pressure sensitive walkway. Vet Surg. (2010) 39:71–7. 10.1111/j.1532-950X.2009.00607.x20210948

[12] ReidJNolanAMScottEM. Measuring pain in dogs and cats using structured behavioural observation. Vet J. (2018) 236:72–9. 10.1016/j.tvjl.2018.04.01329871754

[13] Cimino Brown D. What can we learn from osteoarthritis pain in companion animals? Clin Exp Rheumatol. (2017) 35 (Suppl. 1):53–8.28967360

[14] MeesonRLTodhunterRJBlunnGNukiGPitsillidesAA. Spontaneous dog osteoarthritis - a one medicine vision. Nat Rev Rheumatol. (2019) 15:1. 10.1038/s41584-019-0202-130953036PMC7097182

[15] StadigSLascellesBDXNymanGBerghA. Evaluation and comparison of pain questionnaires for clinical screening of osteoarthritis in cats. Vet Rec. (2019) 185:757. 10.1136/vr.10511531619513PMC6996100

[16] GruenMEGriffithEHThomsonAESimpsonWLascellesBDX Criterion validation testing of clinical metrology instruments for measuring degenerative joint disease associated mobility impairment in cats. Thamm D, editor. PLoS ONE. (2015) 10:e0131839 10.1371/journal.pone.013183926162101PMC4498683

[17] LascellesBDXBrownDCMaixnerWMogilJS. Spontaneous painful disease in companion animals can facilitate the development of chronic pain therapies for humans. Osteoarthr Cartil. (2018) 26:175–83. 10.1016/j.joca.2017.11.01129180098

[18] HercockCAPinchbeckGGiejdaACleggPDInnesJF. Validation of a client-based clinical metrology instrument for the evaluation of canine elbow osteoarthritis. J Small Anim Pract. (2009) 50:266–71. 10.1111/j.1748-5827.2009.00765.x19527419

[19] WaltonMBCowderoyELascellesDInnesJF. Evaluation of construct and criterion validity for the 'liverpool osteoarthritis in dogs' (LOAD) clinical metrology instrument and comparison to two other instruments. Wade C, editor. PLoS ONE. (2013) 8:e58125. 10.1371/journal.pone.005812523505459PMC3591443

[20] MullerCGainesBGruenMCaseBArrufatKInnesJ. Evaluation of clinical metrology instrument in dogs with osteoarthritis. J Vet Intern Med. (2016) 30:836–46. 10.1111/jvim.1392326971876PMC4896092

[21] WaltonBCoxTInnesJ 'How do I know my animal got better?' - measuring outcomes in small animal orthopaedics. Practice. (2018) 40:42–50. 10.1136/inp.k647

[22] BrownDC. The canine orthopedic index. Step 2: Psychometric Testing. Vet Surg. (2014) 43:241–6. 10.1111/j.1532-950X.2014.12141.x24512284

[23] HudsonJTSlaterMRTaylorLScottHMKerwinSC. Assessing repeatability and validity of a visual analogue scale questionnaire for use in assessing pain and lameness in dogs. Am J Vet Res. (2004) 65:1634–43. 10.2460/ajvr.2004.65.163415631027

[24] MinnemaLWheelerJEnomotoMPitakeSMishraSKLascellesBDX. Correlation of artemin and GFRα3 with osteoarthritis pain: early evidence from naturally occurring osteoarthritis-associated chronic pain in dogs. Front Neurosci. (2020) 14:77. 10.3389/fnins.2020.0007732116521PMC7031206

[25] EdwardsSHR. Intra-articular drug delivery: the challenge to extend drug residence time within the joint. Vet J. (2011) 190:15–21. 10.1016/j.tvjl.2010.09.01920947396

[26] LarsenCØstergaardJLarsenSWJensenHJacobsenSLindegaardC. Intra-articular depot formulation principles: role in the management of postoperative pain and arthritic disorders. J Pharm Sci. (2008) 97:4622–54. 10.1002/jps.2134618306275

[27] BannuruRROsaniMCVaysbrotEEArdenNKBennellKBierma-ZeinstraSMA. OARSI guidelines for the non-surgical management of knee, hip, and polyarticular osteoarthritis. Osteoarthr Cartil. (2019) 27:1578–89. 10.1016/j.joca.2019.06.01131278997

[28] ParkKDKimTKBaeBWAhnJLeeWYParkY. Ultrasound guided intra-articular ketorolac versus corticosteroid injection in osteoarthritis of the hip: a retrospective comparative study. Skeletal Radiol. (2015) 44:1333–40. 10.1007/s00256-015-2174-926031217

[29] Osteoarthritis : Care and Management National Clinical Guideline Centre (London) (2020).

[30] KolasinskiSLNeogiTHochbergMCOatisCGuyattGBlockJ 2019 American College of Rheumatology/Arthritis Foundation Guideline for the Management of Osteoarthritis of the Hand, Hip, and Knee. Arthritis Rheumatol. (2020) 72:220–33. 10.1002/art.4114231908163PMC10518852

[31] BruyèreOHonvoGVeroneseNArdenNKBrancoJCurtisEM. An updated algorithm recommendation for the management of knee osteoarthritis from the European Society for Clinical and Economic Aspects of Osteoporosis, Osteoarthritis and Musculoskeletal Diseases (ESCEO). Semin Arthritis Rheum. (2019) 49:337–50. 10.1016/j.semarthrit.2019.04.00831126594

[32] MurrayRCZnaorNTannerKEDeBowesRMGaughanEMGoodshipAE. The effect of intra-articular methylprednisolone acetate and exercise on equine carpal subchondral and cancellous bone microhardness. Equine Vet J. (2010) 34:306–10. 10.2746/04251640277618599412108753

[33] CarterBGBertoneALWeisbrodeSEBaileyMQAndrewsJMPalmerJL. Influence of methylprednisolone acetate on osteochondral healing in exercised tarsocrural joints of horses. Am J Vet Res. (1996) 57:914–22.8725823

[34] ZhangWMoskowitzRWNukiGAbramsonSAltmanRDArdenN. OARSI recommendations for the management of hip and knee osteoarthritis, Part II: OARSI evidence-based, expert consensus guidelines. Osteoarthr Cartil. (2008) 16:137–62. 10.1016/j.joca.2007.12.01318279766

[35] PelletierJ-PMartel-PelletierJ. Protective effects of corticosteroids on cartilage lesions and osteophyte formation in the pond-nuki dog model of osteoarthritis. Arthritis Rheum. (1989) 32:181–93. 10.1002/anr.17803202112920053

[36] RochaRHNatourJdos SantosRMFurtadoRNV. Time effect of intra-articular injection with triamcinolone hexacetonide and its correlations. Am J Phys Med Rehabil. (2019) 98:872–8. 10.1097/PHM.000000000000121731584880

[37] GiganteACallegariL. The role of intra-articular hyaluronan (Sinovial®) in the treatment of osteoarthritis. Rheumatol Int. (2011) 31:427–44. 10.1007/s00296-010-1660-621113807

[38] EvansCH. Novel biological approaches to the intra-articular treatment of osteoarthritis. Biodrugs. (2005) 19:355–62. 10.2165/00063030-200519060-0000316392888

[39] ColenSvan den BekeromMPBellemansJMulierM. Comparison of intra-articular injections of hyaluronic acid and corticosteroid in the treatment of osteoarthritis of the hip in comparison with intra-articular injections of bupivacaine. Design of a prospective, randomized, controlled study with blinding. BMC Musculoskelet Disord. (2010) 11:264. 10.1186/1471-2474-11-26421080920PMC2998460

[40] EvansRHorstmanCConzemiusM. Accuracy and optimization of force platform gait analysis in labradors with cranial cruciate disease evaluated at a walking gait. Vet Surg. (2005) 34:445–9. 10.1111/j.1532-950X.2005.00067.x16266335

[41] StraussEJHartJAMillerMDAltmanRDRosenJE. Hyaluronic acid viscosupplementation and osteoarthritis. Am J Sports Med. (2009) 37:1636–44. 10.1177/036354650832698419168804

[42] SundmanEAColeBJKarasVDella ValleCTetreaultMWMohammedHO. The anti-inflammatory and matrix restorative mechanisms of platelet-rich plasma in osteoarthritis. Am J Sports Med. (2014) 42:35–41. 10.1177/036354651350776624192391

[43] AggarwalASempowskiIP. Hyaluronic acid injections for knee osteoarthritis. Systematic review of the literature. Can Fam Physician. (2004) 50:249–56.15000336PMC2214549

[44] WangC-TLinJChangC-JLinY-THouS-M Therapeutic effects of hyaluronic acid on osteoarthritis of the knee. A meta-analysis of randomized controlled trials. J Bone Joint Surg Am. (2004) 86-A:538–45. 10.2106/00004623-200403000-0001214996880

[45] ChengOTSouzdalnitskiDVroomanBChengJ. Evidence-based knee injections for the management of arthritis. Pain Med. (2012) 13:740–53. 10.1111/j.1526-4637.2012.01394.x22621287PMC3376243

[46] BellamyNCampbellJWelchVGeeTLBourneRWellsGA Viscosupplementation for the treatment of osteoarthritis of the knee. Cochrane Database Syst Rev. (2006) 2006:CD005321 10.1002/14651858.CD005321.pub2PMC888411016625635

[47] SánchezMAnituaEAzofraJAguirreJJAndiaI. Intra-articular injection of an autologous preparation rich in growth factors for the treatment of knee OA: a retrospective cohort study. Clin Exp Rheumatol. (2008) 26:910–3.19032827

[48] ColeBJSeroyerSTFilardoGBajajSFortierLA. Platelet-rich plasma: where are we now and where are we going? Sport Heal A Multidiscip Approach. (2010) 2:203–10. 10.1177/194173811036638523015939PMC3445108

[49] HammondJWHintonRYCurlLAMurielJMLoveringR. Use of autologous platelet-rich plasma to treat muscle strain injuries. Am J Sport Med. (2009) 37:1135–42. 10.1177/036354650833097419282509PMC3523111

[50] NguyenRTBorg-SteinJMcInnisK. Applications of platelet-rich plasma in musculoskeletal and sports medicine: an evidence-based approach. PMR. (2011) 3:226–50. 10.1016/j.pmrj.2010.11.00721402369

[51] AricanMSimşekAParlakKAtliKSönmezG Matrix metalloproteinases 2 and 9 activity after intra-articular injection of autologous platelet-rich plasma for the treatment of osteoarthritis in dogs. Acta Vet Brno. (2018) 87:127–35. 10.2754/avb201887020127

[52] FahieMAOrtolanoGAGuercioVSchafferJAJohnstonGAuJ. A randomized controlled trial of the efficacy of autologous platelet therapy for the treatment of osteoarthritis in dogs. J Am Vet Med Assoc. (2013) 243:1291–7. 10.2460/javma.243.9.129124134578

[53] SilvaRFCarmonaJURezendeCMF. Intra-articular injections of autologous platelet concentrates in dogs with surgical reparation of cranial cruciate ligament rupture. Vet Comp Orthop Traumatol. (2013) 26:285–90. 10.3415/VCOT-12-06-007523612687

[54] AlvesJCSantosAJorgePLavradorCCarreiraLM. A report on the use of a single intra-articular administration of autologous platelet therapy in a naturally occurring canine osteoarthritis model - a preliminary study. BMC Musculoskelet Disord. (2020) 21:127. 10.1186/s12891-020-3140-932106842PMC7047415

[55] CookJLSmithPABozynskiCCKurokiKCookCRStokerAM. Multiple injections of leukoreduced platelet rich plasma reduce pain and functional impairment in a canine model of ACL and meniscal deficiency. J Orthop Res. (2016) 34:607–15. 10.1002/jor.2305426403590

[56] FernándezLChirinoRBoadaLDNavarroDCabreraNdel RioI. Stanozolol and danazol, unlike natural androgens, interact with the low affinity glucocorticoid-binding sites from male rat liver microsomes. Endocrinology. (1994) 134:1401–8. 10.1210/endo.134.3.81191808119180

[57] WrightJKSmithAJCawstonTEHazlemanBL. The effects of the anabolic steroid, stanozolol, on the production of procollagenase by human synovial and skin fibroblasts in vitro. Agents Act. (1989) 28:279–82. 10.1007/BF019674152556901

[58] SpadariARomagnoliNPredieriPGBorghettiPCantoniAMCorradiA. Effects of intraarticular treatment with stanozolol on synovial membrane and cartilage in an ovine model of osteoarthritis. Res Vet Sci. (2013) 94:379–87. 10.1016/j.rvsc.2012.11.02023352201

[59] SpadariARinnovatiRBabbiniSRomagnoliN Clinical evaluation of intra-articular administration of stanozolol to manage lameness associated with acute andchronic osteoarthritis in horses. J Equine Vet Sci. (2015) 35:105–10. 10.1016/j.jevs.2014.12.003

[60] RinnovatiRRomagnoliNSpadariA Dose-finding study for intraarticular treatment with stanozolol in horses. J Equine Vet Sci. (2015) 35:860–4. 10.1016/j.jevs.2015.08.009

[61] MartinsMCPeffersMJLeeKRubio-MartinezLM. Effects of stanozolol on normal and IL-1β-stimulated equine chondrocytes *in vitro*. BMC Vet Res. (2018) 14:1–7. 10.1186/s12917-018-1426-z29554899PMC5859414

[62] PucklerKTellhelmBKirbergerR The hip joint and pelvis. In: Kirberger R, McEvoy F, editors. BSAVA Manual of Canine and Feline Musculoskeletal Imaging. Gloucester: Wiley (2016). p. 212–31.

[63] SmithGKarbeGAgnelloKMcDonald-LynchM Pathogenesis, diagnosis, and control of canine hip dysplasia. In: Tobias K. Johnston S, editors. Veterinary Surgery: Small Animal. 1st ed Saunders (St. Louis, MS). (2011). p. 824–48.

[64] CottaJAiresJMCottaRAntónioDDeJFerreiraA Estudo preliminar para a avaliação da eficácia clínica das infiltrações intra-articulares com estanozolol em canídeos com doença degenerativa articular e a sua relaçõa com a interleucina-1β sérica. University of Lisbon (2016). Available online at: http://hdl.handle.net/10400.5/11299 (accessed June 17, 2018).

[65] Adamama-MoraitouKKPardaliDAthanasiouL VPrassinosNNKritsepiMRallisTS. Conservative management of canine tracheal collapse with stanozolol: a double blinded, placebo control clinical trial. Int J Immunopathol Pharmacol. (2011) 24:111–8. 10.1177/03946320110240011321496393

[66] Van VyncktDSamoyYMosselmansLVerhoevenGVerschootenFVan RyssenB The use of intra-articular anesthesia as a diagnostic tool in canine lameness. Vlaams Diergeneeskd Tijdschr. (2012) 81:290–7.

[67] CaronJP. Intra-articular injections for joint disease in horses. Vet Clin North Am Equine Pract. (2005) 21:559–73. 10.1016/j.cveq.2005.07.00316297721

[68] VolstadNSandbergGRobbSBudsbergS The evaluation of limb symmetry indices using ground reaction forces collected with one or two force plates in healthy dogs. Vet Comp Orthop Traumatol. (2017) 30:54–8. 10.3415/VCOT-16-04-005427849103

[69] PashuckTDKurokiKCookCRStokerAMCookJL. Hyaluronic acid versus saline intra-articular injections for amelioration of chronic knee osteoarthritis: a canine model. J Orthop Res. (2016) 34:1772–9. 10.1002/jor.2319126867692

[70] BrownDCBellMRhodesL. Power of treatment success definitions when the canine brief pain inventory is used to evaluate carprofen treatment for the control of pain and inflammation in dogs with osteoarthritis. Am J Vet Res. (2013) 74:1467–73. 10.2460/ajvr.74.12.146724274882

[71] CarrBJCanappSOMasonDRCoxCHessT. Canine platelet-rich plasma systems: a prospective analysis. Front Vet Sci. (2016) 2:73. 10.3389/fvets.2015.0007326779493PMC4700921

[72] MobasheriAHenrotinY. Identification, validation and qualification of biomarkers for osteoarthritis in humans and companion animals: mission for the next decade. Vet J. (2010) 185:95–7. 10.1016/j.tvjl.2010.05.02620554463

[73] KurokiKCookJLKreegerJM. Mechanisms of action and potential uses of hyaluronan in dogs with osteoarthritis. J Am Vet Med Assoc. (2002) 221:944–50. 10.2460/javma.2002.221.94412369696

[74] ComhaireFHSnapsF. Comparison of two canine registry databases on the prevalence of hip dysplasia by breed and the relationship of dysplasia with body weight and height. Am J Vet Res. (2008) 69:330–3. 10.2460/ajvr.69.3.33018312130

[75] AlvesJCSantosAMJorgePI. Effect of an oral joint supplement when compared to carprofen in the management of hip osteoarthritis in working dogs. Top Companion Anim Med. (2017) 32:126–9. 10.1053/j.tcam.2017.10.00329525231

[76] PsychogiosNHauDDPengJGuoACMandalRBouatraS. The human serum metabolome. PLoS ONE. (2011) 6:e16957. 10.1371/journal.pone.001695721359215PMC3040193

[77] CubukcuDSarsanAAlkanH. Relationships between pain, function and radiographic findings in osteoarthritis of the knee: a cross-sectional study. Arthritis. (2012) 2012:1–5. 10.1155/2012/98406023209900PMC3506881

[78] KhairinaADMoelionoMARahmadiAR Correlation between radiographic grading of osteoarthritis, pain severity and functional status in knee osteoarthritis patients. Althea Med J. (2018) 5:43–6. 10.15850/amj.v5n1.1335

[79] RaynauldJ-PBuckland-WrightCWardRChoquetteDHaraouiBMartel-PelletierJ Safety and efficacy of long-term intraarticular steroid injections in osteoarthritis of the knee: a randomized, double-blind, placebo-controlled trial. Arthritis Rheum. (2003) 48:370–7. 10.1002/art.1077712571845

[80] MendesJGNatourJNunes-TamashiroJCToffoloSRRosenfeldAFurtadoRNV. Comparison between intra-articular Botulinum toxin type A, corticosteroid, and saline in knee osteoarthritis: a randomized controlled trial. Clin Rehabil. (2019) 33:1015–26. 10.1177/026921551982799630782000

[81] WeitoftTÖbergK. Dosing of intra-articular triamcinolone hexacetonide for knee synovitis in chronic polyarthritis: a randomized controlled study. Scand J Rheumatol. (2019) 48:279–83. 10.1080/03009742.2019.157122230843453

[82] CushmanDMOfekESyedRHClementsNGardnerJESamsJM. Comparison of varying corticosteroid type, dose, and volume for the treatment of pain in small- and intermediate-size joint injections: a narrative review. PMR. (2019) 11:758–70. 10.1016/j.pmrj.2018.09.04031166662

[83] PrevitaliDMerliGDi Laura FratturaGCandrianCZaffagniniSFilardoG. The long-lasting effects of “placebo injections” in knee osteoarthritis: a meta-analysis. Cartilage. (2020) 194760352090659. 10.1177/194760352090659732186401PMC8808779

[84] AlvesJCSantosAFernandesÂ. Evaluation of the effect of mesotherapy in the management of back pain in police working dogs. Vet Anaesth Analg. (2018) 45:123–8. 10.1016/j.vaa.2017.07.00629222031

[85] BosscherGTomasARoeSMarcellin-LittleDLascellesBD. Repeatability and accuracy testing of a weight distribution platform and comparison to a pressure sensitive walkway to assess static weight distribution. Vet Comp Orthop Traumatol. (2017) 30:160–4. 10.3415/VCOT-16-09-012828094423

[86] MölsäSHHyytiäinenHKMoreliusKMPalmuMKPesonenTSLappalainenAK. Radiographic findings have an association with weight bearing and locomotion in English bulldogs. Acta Vet Scand. (2020) 62:19. 10.1186/s13028-020-00517-332398017PMC7218547

[87] KennedySLeeDVBertramJEALustGWilliamsAJSoderholmLV Gait evaluation in hip osteoarthritic and normal dogs using a serial force plate system. Vet Comp Orthop Traumatol. (2003) 16:170–7. 10.1055/s-0038-1632773

[88] VassaloFGRahalSCAgostinhoFSMamprimMJMelchertAKanoWT. Gait analysis in dogs with pelvic fractures treated conservatively using a pressure-sensing walkway. Acta Vet Scand. (2015) 57:68. 10.1186/s13028-015-0158-326438541PMC4593187

[89] RiserWHCohenDLindqvistSManssonJChenS. Influence of early rapid growth and weight gain on hip dysplasia in the German Shepherd Dog. J Am Vet Med Assoc. (1964) 145:661–8.5896436

[90] KealyRDLawlerDFBallamJMMantzSLBieryDNGreeleyEH. Effects of diet restriction on life span and age-related changes in dogs. J Am Vet Med Assoc. (2002) 220:1315–20. 10.2460/javma.2002.220.131511991408

[91] InnesJF Arthritis. In: Tobias KM, Johnson SA, editors. Veterinary Surgery: Small Animal. St. Louis: Elsevier Saunders (2012). p. 1078–111.

[92] DouglasRJ. Corticosteroid injection into the osteoarthritic knee: drug selection, dose, and injection frequency. Int J Clin Pract. (2012) 66:699–704. 10.1111/j.1742-1241.2012.02963.x22698422

[93] LabensRMellorDJVoûteLC. Retrospective study of the effect of intra-articular treatment of osteoarthritis of the distal tarsal joints in 51 horses. Vet Rec. (2007) 161:611–6. 10.1136/vr.161.18.61117982139

[94] ZóboliAACde RezendeMUde CamposGCPasqualinTFrucchiRCamargo deOP Ensaio clínico prospectivo e randomizado: regime único e semanal de viscossuplementação. Acta Ortopédica Bras. (2013) 21:271–5. 10.1590/S1413-78522013000500006PMC387499724453681

[95] BaltzerWIOwenRBridgesJ. Survey of handlers of 158 police dogs in New Zealand: functional assessment and canine orthopedic index. Front Vet Sci. (2019) 6:1–6. 10.3389/fvets.2019.0008531058169PMC6478039

[96] OrnettiPNourissatGBerenbaumFSellamJRichettePChevalierX. Does platelet-rich plasma have a role in the treatment of osteoarthritis? Jt Bone Spine. (2016) 83:31–6. 10.1016/j.jbspin.2015.05.00226162636

[97] PopmaJWSnelFWHaagsmaCJBrummelhuis-VisserPOldenhofHGJvan der PalenJ. Comparison of 2 dosages of intraarticular triamcinolone for the treatment of knee arthritis: results of a 12-week randomized controlled clinical trial. J Rheumatol. (2015) 42:1865–8. 10.3899/jrheum.14163026233499

